The article "Lane Detection Algorithm for Intelligent Vehicles in Complex Road Conditions and Dynamic Environments" was published in 2019. Journal: Sensors (Basel).

# Lane Detection Algorithm for Intelligent Vehicles in Complex Road Conditions and Dynamic Environments

**DOI:** 10.3390/s19143166

**Published:** 2019-07-18

**Authors:** Jingwei Cao, Chuanxue Song, Shixin Song, Feng Xiao, Silun Peng

**Affiliations:** 1 State Key Laboratory of Automotive Simulation and Control, Jilin University, Changchun 130022, China; 2 School of Mechanical and Aerospace Engineering, Jilin University, Changchun 130022, China

**Keywords:** driving assistance, intelligent vehicles, edge detection, curve fitting, lane detection

## Abstract

Lane detection is an important foundation in the development of intelligent vehicles. To address problems such as low detection accuracy of traditional methods and poor real-time performance of deep learning-based methodologies, a lane detection algorithm for intelligent vehicles in complex road conditions and dynamic environments was proposed. Firstly, converting the distorted image and using the superposition threshold algorithm for edge detection, an aerial view of the lane was obtained via region of interest extraction and inverse perspective transformation. Secondly, the random sample consensus algorithm was adopted to fit the curves of lane lines based on the third-order B-spline curve model, and fitting evaluation and curvature radius calculation were then carried out on the curve. Lastly, by using the road driving video under complex road conditions and the Tusimple dataset, simulation test experiments for lane detection algorithm were performed. The experimental results show that the average detection accuracy based on road driving video reached 98.49%, and the average processing time reached 21.5 ms. The average detection accuracy based on the Tusimple dataset reached 98.42%, and the average processing time reached 22.2 ms. Compared with traditional methods and deep learning-based methodologies, this lane detection algorithm had excellent accuracy and real-time performance, a high detection efficiency and a strong anti-interference ability. The accurate recognition rate and average processing time were significantly improved. The proposed algorithm is crucial in promoting the technological level of intelligent vehicle driving assistance and conducive to the further improvement of the driving safety of intelligent vehicles.

## 1. Introduction

The annual increase in car ownerships has caused traffic safety to become an important factor affecting the development of a city. To a large extent, the frequent occurrence of traffic accidents is caused by subjective reasons related to the driver, such as drunk, fatigue and incorrect driving operations. Smart cars can eliminate these human factors to a certain extent [1,2,3]. In recent years, the development of smart cars has gradually attracted the attention of researchers in related fields worldwide. Smart cars can intelligently help humans perform driving tasks based on real-time traffic information, thereby indicating their significance in improving the safety of automobile driving and liberating human beings from tedious driving environments [4,5]. Lane detection is an important foundation in the course of intelligent vehicle development that directly affects the implementation of driving behaviours. Based on the driving lane, determining an effective driving direction for the smart car and providing the accurate position of the vehicle in the lane are possible; these features contribute significantly towards improving the efficiency and driving safety of automatic driving [6,7]. Therefore, conducting an in-depth study on this is necessary.

The article "Lane Detection Algorithm for Intelligent Vehicles in Complex Road Conditions and Dynamic Environments" was published in 2019. Journal: Sensors (Basel).

At present, lane detection is mainly based on visual sensors. Visual sensors have essentially become the eyes of a smart car that capture road scenes in front of vehicles through cameras. Such sensors can work continuously for long periods of time with strong adaptability. At the same time, visual sensors have a wide spectrum response range that can see infrared rays, which are invisible to the naked eye; this feature remarkably enlarges the vision space of human beings [8,9,10,11]. However, in daily natural conditions, the problems of vehicle occlusion, insufficient light, varied road twists and turns and complex backgrounds on both sides have caused many difficulties for accurate lane detection [12,13]. With the rapid increase of computer speed, many experts and scholars have focused on lane detection, which is mainly divided into feature- and model-based lane detection. The feature-based lane detection separates the lane from the actual road scene based on the edge and colour features of the lane. Zheng et al. [14] transformed the original RGB image into the CIE colour space and used the adaptive double threshold method to extract the effective features of the lane in the road scene. Haselhoff et al. [15] proposed a method for detecting the left and right lanes by using a two-dimensional linear filter which could eliminate the interference noise during the detection process and preserve the inherent characteristics of the lane in the distant view as much as possible. Son et al. [16] focused on the influence of light changes on lane detection. Based on the illumination invariance of lanes, yellow and white lanes were selected as candidate lanes, and the lanes were also detected via the clustering method from candidate lanes. Amini et al. [17] used the Gabor filter to predict the vanishing point of the lane in the field of vision. When the confidence function was at the maximum confidence level, the line generated below the vanishing point was the lane boundary. In recent years, some experts and scholars have focused on unstructured road detection and curb detection. Kong et al. [18] used vanishing point algorithm to reverse detect road boundary and achieved good results in unstructured road detection. Hervieu et al. [19] used the angle between the normal of the plane fitted with local point data and the ground normal to detect the road boundary, and the Kalman filter model was used to predict the road boundary. The verification results showed that the method was effective for road boundary detection with obstacles. Hata et al. [20] obtained the road boundary points based on elevation jump and slope characteristics, and then discarded the abnormal boundary points by optimization, and finally fitted the road boundary according to the retained boundary points. The model-based lane detection first regards the lane as the corresponding geometric model, and then fits the lane after obtaining the model parameters. Geiger et al. [21] used the Bayesian classifier to obtain the probability generation model based on the pixel points of the road surface and proposed the likelihood function combined with the characteristics of vehicle trajectory and vanishing points. Lane feature recognition was discovered by obtaining the comparative divergence parameters. Liang et al. [22] established an adaptive road geometry model that could analyse the correlation between the road scene ahead and time; hence, the geometry of the lane could be detected and recognised based on the model. Bosaghzadeh et al. [23] solved the problem of obtaining the view angle of the front image by using the principal component analysis (PCA) method. According to the rotation matrix model, lane detection was obtained, and its robustness was acceptable. Recently, deep learning-based methodologies have been used for lane detection. He et al. [24] proposed an algorithm for lane detection based on convolution neural network which converted the input detection image into aerial view. The detection accuracy was high, but the image processing speed was slow and the algorithm took too long. Badrinarayanan et al. [25] proposed SegNet, a pixel-level classification network. Scene segmentation can not only detect lane lines, but also classify and recognize pedestrians, trees and buildings. However, the network had a complicated structure, a large computational load and poor real-time performance. Pan et al. [26] put forward a new neural network Spatial CNN (SCNN) based on visual geometry group, which effectively solved the detection problem when the lane was occluded. The results show that many research methods improved the effective recognition rate of lane detection, but advantages and disadvantages still remain between algorithms that will be limited by various conditions [27,28]. The feature-based lane detection was only applicable to actual road scenes where the lane edges were clear under simple road conditions. When the lane was damaged or visibility was low, the detection accuracy was significantly reduced. In the study of unstructured road detection and curb detection, the accuracy of road boundary detection was high. Nevertheless, when road information was too complicated or there was obstacle interference, the calculation speed was significantly reduced, which easily led to false detection [29,30,31,32]. The model-based lane detection was only suitable for situations in which the preset model was consistent with the detection image and the algorithm must have high complexity and a large calculation amount. In actual road scenes, real-time performance was worse [33,34,35]. Deep learning-based methodologies can effectively improve the accuracy and robustness of lane detection. However, the algorithms had higher hardware requirements, and the training model structures were too complex, so there were still some limitations [36,37,38,39]. Therefore, further improving the lane detection algorithm is necessary.

The article "Lane Detection Algorithm for Intelligent Vehicles in Complex Road Conditions and Dynamic Environments" was published in 2019. Journal: Sensors (Basel).

In this study, a lane detection algorithm for intelligent vehicles in complex road conditions and dynamic environments was proposed. Firstly, converting the distorted image and using the superposition threshold algorithm for edge detection, an aerial view of the lane was obtained by using region of interest (ROI) extraction and inverse perspective transformation. Secondly, based on the curve model, the random sample consensus (RANSAC) algorithm was adopted to fit the curves of lane lines, and the fitting evaluation and the curvature radius calculation on the curve were then carried out. Lastly, by using the road driving video under complex road conditions and the Tusimple dataset, simulation test experiments for lane detection algorithm were carried out. By analysing the experimental results and comparing with other algorithms, the comprehensive performance of the algorithm was evaluated.

The rest of this paper is organised as follows: Section 2 presents the process of converting the distorted image by camera calibration and image distortion removal. Section 3 discusses the edge detection by using the superposition threshold algorithm, and an aerial view of the detection image was obtained via ROI extraction and inverse perspective transformation. Section 4 explains how an effective detection algorithm was used to detect lane lines, and the simulation test experiment based on two datasets and algorithms performance comparison were carried out. Lastly, Section 5 outlines the conclusions and suggests possible future work.

The article "Lane Detection Algorithm for Intelligent Vehicles in Complex Road Conditions and Dynamic Environments" was published in 2019. Journal: Sensors (Basel).

## 2. Converting of Image Distortion

The detection image was captured by a camera mounted on a smart car. Although the camera lens enables the rapid generation of images, such images lead to distortion. In practical terms, distortion changes the shape and size of the lane, vehicle and background in the road scene. These changes are not conducive to judging the correct driving direction and determining the exact location of the vehicle. Consequently, converting of image distortion is essential. In this section, converting of image distortion includes camera calibration and image distortion removal.

### 2.1. Camera Calibration

Instead of focusing on the principle of aperture imaging, the vehicle-mounted camera uses a lens that can focus a large amount of light at one time. These rays bend to varying degrees at the edge of the camera lens and produce the distorted image with edge distortion. The actual road scene is a three-dimensional space, but the collected detection image is a two-dimensional image. Therefore, it was necessary to establish a geometric model between the world and image coordinates and accomplish the camera calibration by obtaining camera characteristic parameters, so as to realize the converting of image distortion.

In the process of describing the geometric relationship of images in the three-dimensional visual space, four coordinates must be defined: World Coordinate *O_w_X_w_Y_w_Z_w_*, Camera Coordinate *O_c_X_c_Y_c_Z_c_*, Image Physical Coordinate *O_1_xy*, and Image Pixel Coordinate *O_o_uv*. Figure 1 illustrates the geometric relationships between coordinates when the image was distorted. Point *p* is the projection point of point *P* on the image plane under the ideal linear model, and point *d* is the projection point of point *P* on the image plane when image distortion occurs.

The two-dimensional image captured by the vehicle-mounted camera must be sequentially converted between the respective coordinates in turn to realise the coordinate transformation of a certain pixel point in the image from the image pixel coordinate to the world coordinate. Figure 2 presents the conversion relationships between the coordinates.

The transformation relationship between the world coordinates of any point P in a three-dimensional space and the image pixel coordinates of the projection point *p* is presented as follows:

(1) $$Z_{c}\left[\begin{array}{c} u\\ v\\ 1 \end{array}\right]=\left[\begin{array}{ccc} \frac{1}{dX} & 0 & u_{0}\\ 0 & \frac{1}{dY} & v_{0}\\ 0 & 0 & 1 \end{array}\right]\left[\begin{array}{cccc} f & 0 & 0 & 0\\ 0 & f & 0 & 0\\ 0 & 0 & 1 & 0 \end{array}\right]\left[\begin{array}{cc} R & t\\ 0^{T} & 1 \end{array}\right]\left[\begin{array}{c} X_{w}\\ Y_{w}\\ Z_{w}\\ 1 \end{array}\right]=\left[\begin{array}{cccc} \frac{f}{dX} & 0 & u_{0} & 0\\ 0 & \frac{f}{dY} & v_{0} & 0\\ 0 & 0 & 1 & 0 \end{array}\right]\left[\begin{array}{cc} R & t\\ 0^{T} & 1 \end{array}\right]\left[\begin{array}{c} X_{w}\\ Y_{w}\\ Z_{w}\\ 1 \end{array}\right]$$

where (*u*_0_, *v*_0_) is the coordinate of point *p* in the Image Pixel Coordinate; *dX* and *dY* are the physical dimensions of each pixel in the Image Pixel Coordinate; *f* is the focal length of the camera; *R* is a unit orthogonal matrix of 3×3 (also called a rotation matrix), which represents the angular relationship between the coordinates; *t* is a translation vector representing the position relationship between the coordinates; (*X_w_, Y_w_*, *Z_w_*) is the homogeneous coordinate of point *p* in the World Coordinate.

The article "Lane Detection Algorithm for Intelligent Vehicles in Complex Road Conditions and Dynamic Environments" was published in 2019. Journal: Sensors (Basel).

Define $\alpha_{x}=f/dX$, which represent the ratio of focal length *f* to the physical dimension of a pixel in the *u*-axis direction. Define $\alpha_{y}=f/dY$, which represent the ratio of focal length *f* to the physical dimension of a pixel in the *v*-axis direction. Then, the above formula can be equivalent to:

(2) $$Z_{c}\left[\begin{array}{c} u\\ v\\ 1 \end{array}\right]=\left[\begin{array}{cccc} \alpha_{x} & 0 & u_{0} & 0\\ 0 & \alpha_{y} & v_{0} & 0\\ 0 & 0 & 1 & 0 \end{array}\right]\left[\begin{array}{cc} R & t\\ 0^{T} & 1 \end{array}\right]\left[\begin{array}{c} X_{w}\\ Y_{w}\\ Z_{w}\\ 1 \end{array}\right]=M_{1}M_{2}\left[\begin{array}{c} X_{w}\\ Y_{w}\\ Z_{w}\\ 1 \end{array}\right]$$

*M*_1_ is a 3×4 matrix determined by parameters such as $\alpha_{x}$, $\alpha_{y}$, *u*_0_ and *v*_0_. These four parameters are related to the internal structure of the camera called the internal parameters of the camera. The rotation matrix *R* and the translation vector *t* are determined by the orientation relationship between the camera and the world coordinates. Therefore, *M*_2_ is called the external parameters of the camera. The internal and external parameters of the camera were obtained through multiple experiments and calculations, and the process of camera calibration was completed.

### 2.2. Image Distortion Removal

In recent years, vehicle-mounted cameras often used wide-angle lens to obtain an enlarged field of vision, and the image distortion changes appeared remarkable. Image distortion is generally divided into radial and tangential distortions. Compared with the actual road scene, the common edge distortion of lanes, vehicles and backgrounds is called radial distortion. If the camera lens is not parallel to the image plane of the visual sensor, the collected image will be tilted, thus making the lane, vehicle and background look closer or farther than in the actual three-dimensional world. This type of image distortion is called tangential distortion, which is more disadvantageous to reflect the real driving environment.

The article "Lane Detection Algorithm for Intelligent Vehicles in Complex Road Conditions and Dynamic Environments" was published in 2019. Journal: Sensors (Basel).

The mathematical model of radial distortion is defined as follows:

(3) $$\left\{\begin{array}{c} u^{\prime }=u(1+k_{1}r^{2}+k_{2}r^{4}+k_{3}r^{6})\\ v^{\prime }=v(1+k_{1}r^{2}+k_{2}r^{4}+k_{3}r^{6}) \end{array}\right.$$

where, *r*^2^ = *x*^2^ + *y*^2^, ($u^{\prime }$,$v^{\prime }$) is the coordinate of point *d* in the Image Pixel Coordinate.

The mathematical model of tangential distortion is presented as follows:

(4) $$\left\{\begin{array}{c} u^{\prime }=u+\left[2p_{1}v+p_{2}(r^{2}+2u^{2})\right]\\ v^{\prime }=v+\left[p_{1}(r^{2}+2v^{2})+2p_{2}u\right] \end{array}\right.$$

Equations (3) and (4) demonstrate that image distortion is related to five parameters—*k*_1_, *k*_2_, *k*_3_, *p*_1_ and *p*_2_—which are collectively called distortion coefficients. By calibrating the camera and acquiring the distortion coefficient, the distorted image can be corrected. In this study, the checkerboard calibration plate was used to remove image distortion. The checkerboard was composed of black and white grids with regular shapes to easily find the coordinates of corner points and observe the image correction conveniently. After determining the coordinates of the corners, a transformation matrix was created to map the distorted points to the undistorted points, and image distortion was removed by using coordinate transformation. Figure 3 shows the correction of the distorted image, in which the left and right halves are the original and undistorted images, respectively.

## 3. Edge Detection and Inverse Perspective Transformation

Edge information is an important feature of the detection image. A suitable edge detection algorithm that can remove a large amount of useless data is beneficial to determine the basic outline of the lane. The inverse perspective transformation converts the detected image into the aerial view to recognise the lane at the optimal visual angle. Therefore, edge detection and inverse perspective transformation are crucial parts in image processing.

### 3.1. Edge Detection

Commonly used edge detection algorithms include global extraction methods based on energy minimisation criterion (such as fuzzy theory and neural networks) and edge derivative methods that use differential operators (such as Canny, Prewitt, LOG and Robert operators). However, the traditional single-edge detection algorithm has many problems, including a too-wide detection range, poor antinoise interference and prolonged calculation time [40,41,42]. Meeting the target requirements of lane detection is difficult. To overcome the shortcomings of the algorithms listed above, this study adopted the edge detection algorithm, which superimposes the threshold of the Sobel operator and HSL colour space.

The article "Lane Detection Algorithm for Intelligent Vehicles in Complex Road Conditions and Dynamic Environments" was published in 2019. Journal: Sensors (Basel).

The Sobel operator is a type of discrete first-order difference operator. The influence of adjacent points in the neighbourhood is different for the current pixel point. Greyscale weighting and differential operations were performed on neighbourhood pixels to obtain the gradient and normal vectors of the pixel point that can be used to calculate the approximate value of the image brightness function.

The Sobel operator performs edge detection on the detected image from the horizontal and vertical directions and can sufficiently filter the interference noise with the improved image processing effect. However, if only the Sobel operator is used for edge detection, then problems such as low detection accuracy and rough edges easily occur. These issues must be solved effectively.

Figure 4 shows the HSL colour space, which can be converted from the common RGB colour space. In this figure, H, S and L denote the hue, saturation and lightness, respectively. H represents the colour change of the image. The position of the spectral colour is represented by the angle, and different colour values correspond to different angles. S refers to the colour degree of the image colour used to describe the similarity between the actual and standard colours. When S is the minimum value of 0, the image becomes a greyscale image and H is undefined. When S is the maximum value of 1, the image colour and its complementary colour are fully saturated. L indicates the lightness degree of the image colour, which gradually changes along the direction of the axis. The maximum and minimum values are 1 and 0 in white and black, respectively.

Compared with the RGB colour space, the HSL colour space can better reflect the visual field perception characteristics of the naked eye. Each colour channel in the HSL colour space can be processed independently and separately. Among them, the component image with S channel performs best and is beneficial to reducing the workload of image processing remarkably and significantly improving the target recognition rate of the detected image.

Gradient threshold segmentation based on the Sobel operator and colour threshold segmentation based on the HSL colour space have advantages and disadvantages. The gradient threshold of the Sobel operator in the *x* direction is superimposed with the colour threshold of the HSL colour space S channel, and the superposition result is shown in Figure 5.

The article "Lane Detection Algorithm for Intelligent Vehicles in Complex Road Conditions and Dynamic Environments" was published in 2019. Journal: Sensors (Basel).

Figure 5a illustrates a threshold superimposition image. To observe the edge detection effects of the two threshold methods intuitively, the gradient threshold segmentation result of the Sobel operator in the *x* direction and the colour threshold segmentation result of the HSL colour space S channel are represented by green and blue, respectively. Figure 5b presents a threshold superimposition binarisation image. By binarising the image, useless interference information can be removed to speed up the operation of the detection algorithm. This figure shows that the edge detection algorithm with threshold superposition achieved good results of complementary advantages and superiorities. These findings are conducive to accurate lane recognition in the detection image and also facilitate the next reverse perspective transformation.

### 3.2. Inverse Perspective Transformation

After edge detection, substantial redundant information, such as the sky, trees and vehicles, still remain in the image. The two-lane lines that appear near-wide and far-narrow gradually meet and make it difficult to detect the lane at a later stage. Therefore, performing ROI extraction and inverse perspective transformation on the detected image is necessary.

#### 3.2.1. ROI Extraction

Given that the vehicle-mounted camera was installed in the middle of the roof of the smart car at a certain depression angle, the detection image contained useless background information, such as the sky, trees and hillsides, on both sides of the road. The effective detection portion, such as the lane, can account for approximately two-thirds of the area of the detected image called ROI. ROI extraction of the detected image can reduce the unnecessary computation and shorten the consumption time of the subsequent image processing step. Figure 6 depicts the extracted ROI.

#### 3.2.2. Inverse Perspective Transformation

Perspective is the phenomenon of images. The closer you get to the camera, the bigger it looks and vice versa. Parallel lane lines merge into a point in the distant field of vision called the vanishing point. The distance between the adjacent lanes near the vanishing point decreases gradually, which is detrimental to effective lane detection. Inverse perspective transformation is based on the inverse coordinate transformation from the world coordinate to the image coordinate that transforms the perspective image into the aerial view and restores the parallel relationship between the lane lines [43,44].

The article "Lane Detection Algorithm for Intelligent Vehicles in Complex Road Conditions and Dynamic Environments" was published in 2019. Journal: Sensors (Basel).

Section 2.1 shows that camera calibration was completed, and the internal and external parameters of the camera were obtained. The internal parameters included focal length and optical centre, whereas the specific external parameters included elevation angle, yaw angle and height of the camera relative to the ground. The inverse coordinate transformation from the world coordinate to the image coordinate was obtained by using Equation (1). Compared with image distortion removal, inverse perspective transformation mapped the position points in the detected image to the new position points in the overlooking perspective to obtain the aerial view of the road image. Figure 7 presents the aerial view of the lane obtained from inverse perspective transformation.

## 4. Lane Detection

Lane detection in complex road conditions is susceptible to external environmental factors, such as lack of light, road tortuosity and vehicle obstruction. The previous image processing was based on a single detection image. However, effective lane detection must be applied in dynamic driving environments while maintaining a recognition rate with sufficiently high accuracy. In this section, the mask operation of the lane was firstly carried out. Then, on the basis of the third-order B-spline curve model, the RANSAC algorithm was used to achieve accurate fitting and curvature calculation of the lane. Lastly, simulation test experiments were performed based on road driving video and the Tusimple datasets, the experimental results were analysed, and the performances of algorithms were compared.

### 4.1. Mask Operation

In the aerial view of the lane, useless interfering pixels still existed. Such interference prolongs not only the image processing time but also easily causes false detection in the next lane detection. Therefore, before lane detection, masking the detected image was necessary. Mask operation essentially filtered the pixel points to highlight the target lane in the detected image.

The mask operation formula is defined as follows:

(5) $$I(i,j)=5\times I(i,j)-\left[I(i-1,j)+I(i+1,j)+I(i,j-1)+I(i,j+1)\right]$$

where I(i,j) is the target pixel point, and I(i−1,j), I(i+1,j), I(i,j−1) and I(i,j+1) are four pixel points around the target pixel. 

Mask operation clearly shows the target pixel point by weighting and averaging the pixels around the target pixel that contributes to sharpening the detection image. Figure 8 shows the detection image after mask operation.

### 4.2. Lane Detection Algorithm

#### 4.2.1. Third-Order B-Spline Curve Model

An *n*-order B-spline curve is defined as

(6) $$\begin{array}{cc} p(t)=\sum_{i=0}^{n}p_{i}B_{i,n}(t) & \left(0\leq t\leq 1\right) \end{array}$$

where $p_{i}(i=0,1,2,\ldots ,n)$ is the position vector of the vertex, and $B_{i,n}(t)$ is the *n*-order basis function presented as follows:

(7) $$B_{i,n}(t)=\frac{n!}{i!(n-1)!}t^{i}{\left(1-t\right)}^{n-i}$$

In the actual road scene, considering that the lane under complicated road conditions tend to be tortuous and variable, the third-order B-spline curve model was used to fit the lane lines. The mathematical expression corresponding to the third-order B-spline curve is as follows:

(8) $$p(t)=p_{0}B_{0,3}(t)+p_{1}B_{1,3}(t)+p_{2}B_{2,3}(t)+p_{3}B_{3,3}(t)$$

By substituting *i* = 0, 1, 2, 3 into Equation (7) separately, the above equation is converted to

(9) $$p(t)=(1-3t+3t^{2}-t^{3})p_{0}+(3t-6t^{2}+3t^{3})p_{1}+(3t^{2}-3t^{3})p_{2}+t^{3}p_{3}$$

This equation is then expressed as the following matrix:

(10) $$\begin{array}{cc} p(t)=\left[\begin{array}{cccc} t^{3} & t^{2} & t & 1 \end{array}\right]\left[\begin{array}{cccc} -1 & 3 & -3 & 1\\ 3 & -6 & 3 & 0\\ -3 & 3 & 0 & 0\\ 1 & 0 & 0 & 0 \end{array}\right]\left[\begin{array}{c} p_{0}\\ p_{1}\\ p_{2}\\ p_{3} \end{array}\right] & \left(0\leq t\leq 1\right) \end{array}$$

where *p*_0_, *p*_1_, *p*_2_ and *p*_3_ correspond to the four control points of the third-order B-spline curve, which can be adjusted accordingly based on real-time road conditions.

The article "Lane Detection Algorithm for Intelligent Vehicles in Complex Road Conditions and Dynamic Environments" was published in 2019. Journal: Sensors (Basel).

#### 4.2.2. Lane Line Fitting Based on RANSAC Algorithm

The RANSAC algorithm is a type of random sampling consistency algorithm. Firstly, random points were obtained from a large number of observation data, and the valid points that met the hypothesis requirements were reserved. The invalid points that failed to meet the hypothesis requirements were discarded. Secondly, the valid points were used to estimate the corresponding models, and the optimal parameters of the estimated model were obtained through continuous iteration. Lastly, the estimation model was accurately fitted based on the obtained effective parameters [45,46].

Figure 9 shows the flow chart for the fitting lane line using RANSAC algorithm.

As can be seen from the above figure, the basic steps for lane line fitting via the RANSAC algorithm are as follows:

(1) Search for the pixel points whose grey value is not equal to 0 in the image to be detected, and the data point set S required by the algorithm is obtained.
(2) According to the third-order B-spline curve model, randomly select four points as the initial valid points of curve fitting in the data point set S, and then an initial third-order B-spline curve is obtained.
(3) Calculate the relative distance between the remaining data points and the initial third-order B-spline curve. Data points that do not exceed the distance threshold *d* are close to the fitting curve, and then the points are added to the valid point set Q as new valid points.
(4) When the number of data points in the valid point set Q reaches the threshold number *n* of the valid points in the preset curve model, step (5) is executed. Otherwise, steps (2) and (3) are repeated until the number of valid points meets the requirements or the upper limit *k* of iteration times is reached.
(5) The third-order B-spline curve is refitted by using the data points in the current valid point set Q, and the best curve fitting result is preserved. When the upper limit *k* of iteration times is reached, the algorithm terminates.

The article "Lane Detection Algorithm for Intelligent Vehicles in Complex Road Conditions and Dynamic Environments" was published in 2019. Journal: Sensors (Basel).

The RANSAC algorithm can reduce the interference of invalid points in curve fitting, and the curve model can be re-estimated by the continuous accumulation of valid points. With the increasing number of iterations, the obtained fitting curve gradually tends to be the best and minimises the error between the fitting curve and the real lane line. The RANSAC algorithm based on the third-order B-spline curve model was used to fit the lane lines. This algorithm can describe lane lines with different shapes and has good adaptability and robustness.

Figure 10 presents the lane line fitting result.

#### 4.2.3. Lane Line Fitting Evaluation and Curvature Radius Calculation

The RANSAC algorithm uses the continuous iterative method to obtain the optimal fit curve. Therefore, determining an effective evaluation criterion for lane line fitting is necessary. The comparison of the error rate magnitude between the fitting curve and the real lane line determines the best lane line fitting result. 

When the distance from all valid points in the area around the fitting curve to the fitting curve was the smallest, the error between the fitting curve and the real lane line was minimised, and the lane line fitting evaluation score was the highest. The following evaluation score (*Score*) is defined as the reciprocal of the mean of the relative distance between all data points in the valid point set Q and the fitting curve:

(11) $$Score=\frac{n}{\sum_{i=1}^{n}\left|{\left(x_{t}\right)}_{i}-{\left(x_{sp}\right)}_{i}\right|}$$

where i=0,1,2,…,n, and *n* is the number of all data points in the valid point set Q.

The curvature of the current lane line was used to express its curve degree. The reciprocal of the curvature is the curvature radius, which was used in this study to represent the curvature (in *m*). The curvature calculation of the third-order B-spline curve is more complicated than that of the simple curve. In this study, the original curve was reduced in order, the first and second derivative curves re-obtained by first- and second-order reduction, respectively. In the two-dimensional plane, let the coordinate corresponding to the first derivative be $(x^{\prime },y^{\prime })$ and the coordinate corresponding to the second derivative be $\left(x^{\prime \prime },y^{\prime \prime }\right)$. The curvature of the lane line is defined as follows:

(12) $$K=\frac{x^{\prime }y^{\prime \prime }-y^{\prime }x^{\prime \prime }}{{\left[{\left(x^{\prime }\right)}^{2}+{\left(y^{\prime }\right)}^{2}\right]}^{3/2}}$$

Figure 11 illustrates the lane line detection result of the detected image. The left and right lane lines were detected, and the corresponding evaluation scores were obtained based on their valid points. The curvature and average curvature radii of the left and right lane lines were calculated (the specified curve is positive and negative in the clockwise and counterclockwise directions, respectively). 

The article "Lane Detection Algorithm for Intelligent Vehicles in Complex Road Conditions and Dynamic Environments" was published in 2019. Journal: Sensors (Basel).

### 4.3. Simulation Test Experiment

#### 4.3.1. Test Environment

Software environment: Windows 10 64-bit operating system, Python 3.7.0 64-bit, OpenCV 4.1.0, FFMPEG 1.4.

Hardware environment: Intel (R) Core (TM) i5-6500 CPU@3.20GHz processor, 8.00 GB memory, 2 TB mechanical hard disk.

#### 4.3.2. Lane Detection Based on Road Driving Video

To verify the recognition performance of the lane detection algorithm in complex working conditions and dynamic environments, road driving videos were used to carry out the simulation test experiment in this work. Such videos in the experiment were collected by using a real-time vehicle-mounted camera, and the lane lines were detected for different road conditions, such as highway, mountain road and tunnel road.

Furthermore, the classical sliding window search method was utilised to test the lane detection algorithm dynamically in the simulation test experiment. Firstly, a pixel histogram was generated by the pixels whose grey value was not equal to 0, and the peak value in the pixel point set was obtained (the area where the lane line exists). Secondly, the sliding window was used to accumulate from bottom to top. When the number of pixels in the window exceeded the set threshold number, the mean value was taken as the centre of the next sliding window. In addition, by using the sliding window search method, the offset of the vehicle relative to the centre position of the road could be estimated.

Figure 12, Figure 13, and Figure 14 illustrate the lane line detection results under complex road conditions respectively.

Figure 12 shows the test result of a typical detected frame in the highway driving video. The figure intuitively demonstrates that the proposed algorithm could still accurately detect the left and right lane lines although the speed of the vehicle on the highway is fast. Compared with other road conditions, the curve degree of the lane line was the smallest, the curvature radius was the largest and the corresponding sliding window offset was the smallest. Figure 13 shows the test result of a typical detected frame in the tunnel road driving video. The figure intuitively shows that the proposed algorithm could still accurately detect the left and right lane lines although the lighting conditions on the tunnel road were poor. Compared with highway conditions, the curve degree of the lane line was larger, the curvature radius was smaller and the corresponding sliding window offset was larger. Figure 14 depicts the test result of a typical detected frame in the mountain road driving video. The figure intuitively presents that the proposed algorithm could still accurately detect the left and right lane lines although the mountain road was tortuous and changeable with many trees on both sides of the road. Compared with other road conditions, the curve degree of the lane line was the largest, the curvature radius was the smallest and the corresponding sliding window offset was the largest.

The article "Lane Detection Algorithm for Intelligent Vehicles in Complex Road Conditions and Dynamic Environments" was published in 2019. Journal: Sensors (Basel).

Table 1 lists the lane detection results based on road driving video under complex road conditions.

In the lane detection test experiment, the accurate recognition rate under highway condition reached 99.15%, and the average processing time per frame was 20.8 ms, thereby indicating that the lane detection algorithm had good real-time performance and accuracy. The accurate recognition rate under tunnel road condition reached 98.47%, and the average processing time per frame was 21.6 ms, thereby indicating that the lane detection algorithm still had good adaptability in case of insufficient light. The accurate recognition rate under mountain road condition reached 97.82%, and the average processing time per frame was 22.1 ms, thus indicating that the lane detection algorithm still had good robustness and antijamming ability in the case of road tortuosity and background interference. 

By sorting and analysing false or missed detection images, the majority of these images were caused by motion blur, vehicle occlusion, insufficient light and excessive road bending. In the future, improving the lane detection algorithm will be necessary to enhance its complexity and efficiency. Collecting road traffic videos with varied road conditions will also be important to improve the inclusiveness and robustness of the lane detection algorithm continuously.

The article "Lane Detection Algorithm for Intelligent Vehicles in Complex Road Conditions and Dynamic Environments" was published in 2019. Journal: Sensors (Basel).

#### 4.3.3. Lane Detection Based on the Tusimple Dataset

In order to further test the comprehensive performance of the proposed algorithm under a variety of complex road conditions, in addition to the road driving videos for simulation test experiments, the Tusimple dataset (general-purpose benchmark dataset) was also used for lane detection. The Tusimple dataset consists of 3626 training images and 2782 testing images, and each sequence image comprising 20 consecutive frames taken in 1s, of which the first 19 frames are unmarked and the 20th frame is labelled with lane ground truth. The images in the dataset can be roughly divided into four conditions, including different weather conditions, daytime, lanes number (2 lanes/3 lanes/4 lanes or more), and traffic environments [47,48]. 150 images representing different conditions were randomly extracted from the Tusimple dataset separately in this work, and the lane detection experiments were carried out using the proposed algorithm.

Figure 15 shows the lane detection results under different typical conditions.

Table 2 lists the lane detection results under different conditions in the Tusimple dataset.

It can be seen from Figure 15 and Table 2 that the proposed algorithm worked well under different conditions in the Tusimple dataset. In the statistics of lane detection results in four different conditions, the test accuracy was the highest under different lanes number conditions, the accurate recognition rate was 99.13%, and the average processing time per frame was 22.8 ms. The test accuracy was the lowest under different traffic environment conditions, but the accurate recognition rate also reached 97.70%, and the average processing time per frame was 22.5 ms. In total, the average accurate recognition rate under four different conditions reached 98.42%, and the average processing time per frame was 22.2 ms. Compared with the results of lane detection in the road driving video, the average accurate recognition rate was slightly reduced, and the average processing time per frame was also slightly extended. However, the proposed algorithm still has good comprehensive recognition performance in the Tusimple dataset, thus indicating desirable accuracy and adaptability.

### 4.4. Algorithms Performance Comparison

To verify the performance of the lane detection algorithm, the proposed algorithm was compared with other algorithms used in the literature. Table 3 lists the comparison of statistics in algorithms performance.

In this paper, the proposed algorithm was compared with traditional detection methods and deep learning-based methodologies. In particular, the proposed algorithm and reference [51] and [52] all carried out relevant lane detection test experiments based on the Tusimple dataset. In reference [49], the feature-based lane detection method was adopted. Compared with other algorithms, although the average processing time was relatively short, the average detection accuracy was the lowest and more likely to cause false or missed detection in actual road scenes. In Reference [50], the model-based lane detection method was adopted. Compared with literature [49], although the average detection accuracy did improved, the average processing time was too long. When this algorithm was applied to actual road scene, the problem of poor real-time performance existed. In Reference [51], the lane structure was predicted relevantly by training FastDraw Resnet, and the proposed method was tested effectively based on the CVPR 2017 Tusimple lane marking challenge, difficult CULane datasets. Compared with traditional detection methods, this method achieved higher recognition accuracy, and the values of FP and FN were kept at a lower level, reflecting the competitive advantage of deep learning-based methodologies. In Reference [52], lane detection was performed using the ConvLSTM network model based on the Tusimple dataset and their own lane datasets. Compared with literature [51], the recognition accuracy was further improved, the average processing time was further shortened, and the values of FP and FN were significantly reduced, thus reflecting good robustness and stability. However, due to the complex structure of the training model and the large calculation amount of the algorithm, deep learning-based methodologies were prone to problems such as too long training time and poor real-time performance, and there is still room for further improvement. Compared with literature [51] and [52], the proposed algorithm achieved the best overall performance with the same data set, the average accurate recognition rate reached 98.42%, and the average processing time per frame was 22.2 ms. In terms of performance improvement, it had obvious advantages. The fully improved lane recognition accuracy was conducive to greatly enhancing the driving safety of intelligent vehicles in the actual driving environments, and the fully shortened average processing time was conducive to effectively meeting the real-time target requirements of intelligent vehicles in the actual driving environments, and stable detection under complex working conditions and dynamic environments was conducive to improving the anti-interference ability and environmental adaptability of intelligent vehicles as a whole, thus contributing to further improving the technical level of intelligent vehicle driving assistance.

The article "Lane Detection Algorithm for Intelligent Vehicles in Complex Road Conditions and Dynamic Environments" was published in 2019. Journal: Sensors (Basel).

## 5. Conclusions

This study proposed a lane detection algorithm for intelligent vehicles in complex road conditions and dynamic environments. Firstly, converting the distorted image and using the superposition threshold algorithm based on the Sobel operator and HSL colour space for edge detection, an aerial view of the lane was obtained by using ROI extraction and inverse perspective transformation. Secondly, the RANSAC algorithm was adopted to fit the curves of the lane lines on the basis of the third-order B-spline curve model, and the fitting evaluation and the curvature radius calculation on the curve were carried out next. Lastly, by using the road driving video under complex road conditions and the Tusimple dataset, simulation test experiments for lane detection algorithm were performed. The experimental results show that the average detection accuracy based on road driving video reached 98.49%, and the average processing time reached 21.5 ms. The average detection accuracy based on the Tusimple dataset reached 98.42%, and the average processing time reached 22.2 ms. Compared with traditional methods and deep learning-based methodologies, this lane detection algorithm had excellent accuracy and real-time performance, high detection efficiency and strong anti-interference ability. The accurate recognition rate and average processing time were significantly improved.

In terms of lane detection accuracy and algorithm time-consuming, the proposed lane detection algorithm had clear advantages. It was conducive to greatly enhancing the driving safety of intelligent vehicles in the actual driving environments and effectively meeting the real-time target requirements of smart cars and played an important role in intelligent vehicle driving assistance. In the future, the inclusiveness and anti-error detection of the lane detection algorithm can be further optimised and improved to exploit the overall performance of the algorithm.

## Figures and Tables

**Figure 1:** The geometric relationships between coordinates when the image is distorted.

**Figure 2:** The conversion relationships between the coordinates.

**Figure 3:** The correction of the distorted image.

**Figure 4:** The HSL colour space.

**Figure 5:** Gradient threshold and colour threshold superposition result.

**Figure 6:** The extracted ROI.

**Figure 7:** The aerial view of the lane.

**Figure 8:** The detection image after mask operation.

**Figure 9:** Flow chart for fitting lane line using the random sample consensus (RANSAC) algorithm.

**Figure 10:** The lane line fitting result.

**Figure 11:** The lane line detection result.

The article "Lane Detection Algorithm for Intelligent Vehicles in Complex Road Conditions and Dynamic Environments" was published in 2019. Journal: Sensors (Basel).

**Figure 12:** The test result of a typical detected frame in the highway driving video.

**Figure 13:** The test result of a typical detected frame in the tunnel road driving video.

**Figure 14:** The test result of a typical detected frame in the mountain road driving video.

**Figure 15:** The lane detection results under different typical conditions.

**Table 1:** The lane detection results based on road driving video under complex road conditions.

Video Sequence Number	Complex Road Conditions	Total Frames	Detected Frames	Misdetected and Missed Frames	Accurate Recognition Rate (%)	Average Processing Time (ms)/ Frame
1	Highway	1535	1522	13	99.15	20.8
2	Tunnel Road	1763	1736	27	98.47	21.6
3	Mountain Road	1470	1438	32	97.82	22.1
Total	-	4768	4696	72	98.49	21.5

**Table 2:** The lane detection results under different conditions in the Tusimple dataset.

Sequence Number	Condition Type	Lanes Total Number	Correct Recognition Number	False and Missed Recognition Number	Accurate Recognition Rate (%)	Average Processing Time (ms)/ Frame
1	Weather	573	561	12	97.91	21.9
2	Daytime	561	555	6	98.93	21.7
3	Lanes Number	578	573	5	99.13	22.8
4	Traffic Environment	566	553	13	97.70	22.5
Total	-	2278	2242	36	98.42	22.2

**Table 3:** The comparison of statistics in algorithms performance.

Method	Algorithm	Average Detection Accuracy (%)	Average Processing Time (ms)/ Frame	FP	FN	System Environment
Traditional	Spatial Ray Features [49]	94.40	45.0	-	-	NVIDIA GeForce GTX 580, GPU
	Improved Hough Transform [50]	95.70	65.4	-	-	Intel Core i7-6700K CPU @ 4 GHz
Deep Learning	FastDraw Resnet [51]	95.00	65.3	0.065	0.048	NVIDIA GeForce GTX 1080, GPU
	ConvLSTM [52]	97.25	42.0	0.042	0.0185	Intel Core Xeon E5-2630 @ 2.3 GHz, GeForce GTX TITAN-X GPU
Proposed	Ours	98.42	22.2	-	-	Intel(R) Core(TM) i5-6500 CPU @ 3.20 GHz
